This article has been retracted.

# Performance Evaluation of Hospital Economic Management with the Clustering Algorithm Oriented towards Electronic Health Management

**DOI:** 10.1155/2022/3603353

**Published:** 2022-04-06

**Authors:** Tian Tian, Dixin Deng

**Affiliations:** ^1^Youth League Committee, The First Affiliated Hospital, University of South China, Hengyang 421001, Hunan, China; ^2^Finance Department, The First Affiliated Hospital of University of South China, Hengyang 421001, Hunan, China

## Abstract

In order to study the clustering algorithm based on density grid, the performance evaluation index system of hospital economic management under the application of electronic health management system is constructed. Firstly, this work designs the basic architecture of electronic health management system, classifies and screens the process of index system of electronic health management system, compares the clustering algorithm based on density grid with the simple clustering algorithm based on density or grid, and then applies it to the performance evaluation index system of hospital economic management. According to the principle of Mitchell scoring method, the expert questionnaire of hospital economic management performance evaluation index system was designed, and Delphi method was used to evaluate the candidate indexes from the three dimensions of right, legitimacy, and urgency. The results show that, compared with simple network clustering algorithm and density clustering algorithm, the clustering algorithm based on density network produces higher purity (94% VS 73% VS 67%) and lower entropy (0.9 VS 1.4 VS 1.54), which effectively saves memory consumption, and the difference is statistically significant (*P* < 0.05). The core indicators with scores above 4.5 in both dimensions include budget revenue implementation rate, budget expenditure implementation rate, implementation rate of special financial appropriation, asset-liability ratio, hospitalization income cost rate, medical insurance settlement rate, average cost of discharged patients, and drug proportion. The coefficient of variation of the first grade index is between 0.05 and 0.14 and that of the second grade index is between 0.05 and 0.15. Clustering algorithm based on density network has higher purity and lower entropy, which can effectively save memory consumption. The performance evaluation index system of hospital economic management finally determines 6 first-level indexes: budget management, financial fund management, cost management, medical expense management, medical efficiency, medical quality, and 25 second-level indexes.

## 1. Introduction

In the era of big data today, the public social activities on the Internet become continuous and comprehensive gradually, and more and more people are willing to upload personal health information to the cloud. Electronic health management has become a key social issue. In recent years, new network information technology has been mainly developed on artificial intelligence, databases, and fifth-generation (5G) networks, and the rudiment of a complex and comprehensive digital society has been gradually shown. Therefore, the development of electronic health management becomes an inevitable phenomenon [1–3]. A latest survey report released by the Global Web Index (GWI) shows that social media users account for 98% of global Internet users. With the ever-increasing social media users, people face with the biggest opportunity and challenge of information disclosure globally in the personal electronic health management. In some developed countries, such as the United States, the United Kingdom, and Japan, the management of personal health information is stressed, and the specific protective laws have been issued. There is a similar history of information protection laws in electronic health management in these countries, all of which show a transition from the health information protection to the construction of a health information system [4–7]. China is an important economic entity in the world, but there are still many shortcomings in the laws on electronic health management. The personal health information cannot be protected essentially, as it mainly relies on relevant laws. In addition, the needs of some institutions for electronic health management cannot be satisfied due to the lack of effective laws. It is necessary to resolve the conflict reasonably between the public needs for electronic health management and its safety and keep the balance between the relevant institutions and the public needs, for the stable development of society and the improvement of the electronic health management.

The Guidelines on the Establishment of a Modern Hospital Management System of the General Office of the State Council (No. 67 [2017]) was issued by the General Office of the State Council on July 14, 2017, pointed out that the establishment of a comprehensive hospital management system can be started with the financial asset management system and the performance assessing system. The *Guidelines on Strengthening the Operation and Management of Public Hospitals* (No. 27 [2020]) was issued by the National Health Commission on December 25, 2020. It was stated that it is necessary to accelerate the transformation of management model and operating mechanism to promote the high-quality development of public hospitals so that the hospitals could meet the scientific, refined, and informatized standard and meet the relevant requirements of the public hospital operation and management system. The most important thing in the reform of public hospitals is to improve the hospital economic management comprehensively. The public hospital reform can be reflected through changes in the economic management [8–10]. In addition, for comprehensive improvement of the economic management of hospitals, it is required to innovate the operating mechanism of public hospitals and improve the financial management system and economic operation system. The hospital economic management is mainly reflected in its performance evaluation, and the feasibility of performance plan depends on the performance evaluation indicator system of hospital economic management.

Hospital economic management refers to the strengthening of hospital economic activities with economic means in accordance with objective laws of economic development, through improving hospital management systems and hospital management methods continuously [11, 12]. Manpower, property, and resources should be reasonably used to reduce labour costs as much as possible, and the medical and health service technology should also be continuously improved to achieve the greatest economic outcome. Thus, the healthcare-centred teaching and research could be better completed and the increasing medical needs of people could be satisfied. Performance evaluation refers to a comprehensive evaluation of the implementation degree and results of hospital management goals, using specific evaluation methods with the evaluation standards and quantitative indicators. Ohio University Research puts forward two aspects, including internal evaluation and external evaluation, as the overall framework of performance measurement of medical and health institutions, each of which includes two dimensions of financial performance and quality performance [13]. Sana mentioned that the hospital performance management system mainly includes three aspects: first, the management analysis, the implementation of branch management in hospitals, daily analysis and comparison of operating results, and regular review. Second, the quantity can be checked, and all personnel have a reward mechanism. Third, personnel management, the labour cost accounts for about half of the total hospital cost, and poor personnel management will cause adverse effects [14]. With the issuance of Bitcoin, blockchain, the underlying core technology of the Bitcoin system has gradually come into people's life as a database technology with the advantages of openness, flatness, and equality. Blockchain technology takes the trust security as the core, not only innovating the pattern of traditional Internet but also promoting efficient operation in transactions, authentication, and other aspects. Blockchain technology can also promote the synergy of multiple energies and various participating entities, the rapid integration of information and physical systems, the diversification of transactions, and cost minimization. Data mining is an interdisciplinary subject including artificial intelligence, pattern recognition, statistics, database, and neural network, including prediction verification function and description function. Among them, the prediction verification function includes association analysis, sequence pattern mining, and regression analysis. Functions include classification, clustering, feature analysis, and deviation analysis. The team led by the professor of Stanford University focuses on data stream management, continuous query, and clustering. Clustering algorithm is an important data mining method, which divides an object set into several clusters according to some similarity measure criterion, and the objects in the same cluster have high similarity in some aspects. The purpose of clustering algorithm is to divide a data set into unconnected clusters with the same attributes. Clustering algorithm is widely used, and it has been developed in many fields such as commerce, medical care, geography, insurance industry, Internet application, and e-commerce [15–21]. Combining the advantages of the density-based and the grid-based clustering algorithms, the clustering algorithm is an important data mining method, which divides an object set into several clusters according to some similarity measure criterion, and the objects in the same cluster have high similarity in some aspects. Grid-based algorithm is a clustering algorithm based on multiresolution idea, which divides the data sample space into a limited number of cells to form a grid structure, and finally all clustering operations are carried out on the grid. The main advantage of this method is that the processing speed is fast, and the clustering process is independent of the number of original data samples and only depends on the maximum number of grid cells. Combining the advantages of density-based clustering algorithm and grid-based clustering algorithm, this study uses density-grid-based clustering algorithm to cluster data samples and uses blockchain technology to apply it to hospital economic management performance evaluation system and achieves ideal results.

At present, academic performance evaluation in different fields has achieved remarkable results, but there is no sufficient theoretical support for hospital economic management performance evaluation under electronic health management [22]. Extensive economic management generally exists in public hospitals, which directly affects the overall operation effect of the hospital. In order to maintain the normal survival and development of the hospital, hospital managers increase hospital revenue by constantly expanding the scale of the hospital, adding large-scale equipment and increasing charging items. Although this relieves the pressure of the hospital to a certain extent, the algorithm still covers up the real situation of poor internal management of the hospital, which is not conducive to the self-adjustment and improvement of hospital management direction, and at the same time, it harms the interests of patients to a certain extent. From the perspective of economic management, this work formulates the performance evaluation index system of hospital economic management, which is beneficial to the hospital to clarify the key points of economic management, adjust the development of operation mode from extensive to refined, and enable the hospital construction to enter the benign track of sustainable development, thus fully reflecting the value orientation of public welfare, efficiency, and fairness of public hospitals, meeting the medical needs of the broad masses of people and completing other related tasks of public hospitals.

## 2. Technologies and Methods

### 2.1. Basic Architecture of the Electronic Health Management System

The basic architecture of the management platform mainly included the host terminal structure, client/server (C/S) structure, browser/server (B/S) structure, and file server structure. With the development of the network computing and the rapid increase of social media users, the B/S structure gave a highly stable technical platform with C/S structure. The B/S structure itself had diversified modes, and its client was a very convenient browser, while the server was responsible for complex data processing. The major advantage of the B/S structure was the convenient configuration of the client, which was conducive to the development and maintenance of the system.

Client users could complete the information publishment through simple and flexible operations. In this study, a three-tier B/S structure was taken as the development tool for the basic architecture design. The first tier was the client, mainly providing basic services for doctor workstations and individual users. The second tier was the application server to operate the business processing of the hospital system with two servers. The data storage, replacement, management, and other operations could be done through the tier. The third tier was the data tier consisting of database and other systems, and it was designed for the storage and management of information data. The architecture is shown in Figure 1.

According to the main business steps of electronic health management, the flow of health data information was taken as the major direction of system operation, and the preliminary software framework of electronic health management system was designed. The framework included 5 main parts, which were data collection and transmission, health check, health risk assessment, automatic intervention measures, and interfaces, as shown in Figure 2.

### 2.2. Construction Process of Electronic Health Management Index System

At the initial stage of the index system construction, it is necessary to collect relevant literature materials of health information management and performance evaluation to provide theoretical support for the establishment of electronic health management index evaluation index system. Through on-the-spot investigation, questionnaire survey, symposium, and other forms, it can understand the development of medical services, investigate the situation of health information management in depth, and build the performance evaluation index system of health information management. To construct the performance evaluation index system of health information management, relevant principles should be followed, and scientific evaluation methods should be selected to construct it. At this stage, different standards should be set for the main contents that affect the performance of health information management, the factors that affect health information management should be refined and quantified, and the relevant weights should be determined. In order to test the rationality of the health information management performance evaluation index system, it is necessary to optimize and test it. Finally, after passing the relevant tests, before formally establishing the performance evaluation index of health information management, actual testing is a necessary procedure to ensure the operability of the index system, and the established index system is revised through the test results, as shown in Figure 3.

### 2.3. Blockchain Technology

Blockchain network is a point-to-point network. The whole network has no centralized hardware structure (central server) and management mechanism (central router). Each node in the blockchain network has equal status and can be used as both a client and a server. Each node retains all data resources of the entire blockchain network, and all network data have multiple backups. The more the nodes participating in the network, the more the data backup. In the prior art, the backup of blockchain is completed by each node by itself, and when the backup conditions are met, the blockchain node uploads data to the designated server, which may result in repeated backup, wasting network, and server resources, and the backup efficiency is not high. On the other hand, in the prior art, backup information needs to be maintained by blockchain nodes or blockchain networks themselves, which also brings a burden to blockchain networks and wastes resources, and self-maintenance of backup information will also lead to security problems of backup information. Therefore, this study optimizes the backup method of blockchain data so that each node can enter or leave the network at will to maintain the stability of the network. In addition, the possibility of data modification is reduced.

In the encryption system of blockchain network, an asymmetric encryption algorithm was adopted to deal with the trust issue among network users. The asymmetric encryption algorithm is run with two types of keys: the public key and a private key, which were matched one to one. As the public key was used to encrypt the processed data, only the matched private key could decrypt it. In the same way, if the processed data were encrypted through the private key, only the corresponding public key could decrypt it. Each user in the blockchain had a unique public key and private key, of which the public key was public to all users on the network. Users on the blockchain network used the same encryption algorithm, and the private key was owned by its user alone. The user encrypted the information with the private key, and other users could decrypt the information with the public key.

### 2.4. Operating Environment of the Electronic Health Management System

The server adopted Windows 10.0 operating system, and it was more advanced than Microsoft SQL2005. The processor was of P4 3.0 GHz, and the hard disk capacity was 120G. The Windows 10.0 operating system was also adopted for the client with Microsoft Office 2013; the P4 3.0 GHz processor and the 1920 × 1080 resolution of display screen were applied as well.

### 2.5. The Density-Grid Clustering Algorithm

In the density-grid clustering algorithm, the density threshold of grid cells was generally used to distinguish dense grid cells from sparse grid cells. Then, the neighbouring dense grid cells were merged into a grid cluster to achieve the clustering effect. Thus, the parameters of the density threshold affected the clustering results directly. If the density threshold was set too small, the algorithm might not be able to distinguish the dense areas from sparse areas accurately in the data space. There would be a lot of noises in the final clustering results obtained, which reduced the quality of clustering. If it was set too large, the algorithm would recognize a large number of evenly distributed clusters as sparse grid cells. Even in the Gaussian distributed clusters, only a few high-density independent grid cells could be found [23]. The idea of mean density was adopted in this study, so part of the data was collected for the statistics of data density distribution, and then the grid cell density threshold of the algorithm was determined with the basic statistical information.

In the process of data flow processing, *N*, the amount of data in the network unit, is firstly, and then grid cells with the data are counted to calculate the maximum value *U*_max_, mean value *U*_mean_, and minimum value *U*_min_ of the cell density.

The equation for the mean value of network cell density is as follows:

(1) $$\begin{array}{c} U_{\text{mean}}=\frac{\sum_{i=1}^{N}U_{i}}{N}. \end{array}$$

In (1), *U*_*i*_ represents the density of the network cell density *f*, and *N* is the number of network grid cells.

The dense grid cell threshold is computed through

(2) $$\begin{array}{c} U_{d}=\frac{U_{\max}+U_{\text{mean}}}{2}. \end{array}$$

In (2), *U*_*d*_ stands for the dense grid cell threshold and *U*_max_ and *U*_mean_ are the maximum value and the mean value of the network cell density, respectively.

The sparse grid cell threshold is calculated via

(3) $$\begin{array}{c} U_{s}=\frac{U_{\text{min}}+U_{\text{mean}}}{2}. \end{array}$$

In (3), *U*_*s*_ is the sparse grid cell threshold, and *U*_min_ represents the maximum value of the cell density.

At some time, the mean density of clusters in the data flow is very high, but it may change to be very low at the next moment. It means that the density of clusters in the data flow is changing constantly over time.

As time goes by, new data samples in the data flow would be input into the computer system continuously and mapped to the corresponding data unit. If the dense grid cell had not received new data samples for a long time, it might degenerate into a sparse grid. On the contrary, if the sparse grid cell received a batch of new data samples in a certain period of time, it might be upgraded to a dense grid [24–26]. Therefore, it was necessary to monitor the network density regularly and the clusters that had been generated should also be adjusted. The grid density detection period (*P*) was related to the clustering result directly, so it cannot be too long or too short.

**Theorem 1 .**

The minimum time required for a dense grid to degenerate into a sparse grid is represented as Δ*T*_min_^−^, which is calculated by the following

(4) $$\begin{array}{c} \Delta T_{\text{min}}^{-}=\frac{1}{\gamma }\log\frac{\delta }{\delta -1}. \end{array}$$

In (4), the parameter *δ* is the density threshold, and *δ* > 0; and 0 < *γ* < 1.

**Theorem 2 .**

The minimum time required for a sparse grid to be upgraded into a dense grid is Δ*T*_min_^+^, which is expressed as

(5) $$\begin{array}{c} \Delta T_{\text{min}}^{-}=\left|\frac{1}{\gamma }\log\frac{G\left(f,t\right)\left(1-2^{-\delta }\right)-1}{\delta \left(1-2^{-\delta }\right)-1}\right|. \end{array}$$

In (5), *G*(*f*, *t*) represents the density of grid cell *f* at *t*; *δ* is the density threshold, and *δ* > 0; and 0 < *γ* < 1. The density detection period *P* should be the smallest integer between Δ*T*_min_^−^ and Δ*T*_min_^+^.

**Proof**

Assuming that grid element *f* is a sparse grid, it is upgraded to a dense grid after time Δ*T*. Therefore, because of the set *S*(*f*, *t*)⊆*S*(*f*, *t*+Δ*T*), the data samples of *S*(*f*, *t*+Δ*T*) in the set can be divided into two categories: one is the data sample points of the set *S*(*f*, *t*), and the other is the data samples that arrive between time *t* and time *t*+Δ*T*. The necessary condition for a sparse grid *F* to be upgraded to a dense grid is that all data samples arriving between *t* and *t*+Δ*T* are mapped to the *F* grid. This means that from the time of *t* and *t*+Δ*T*, a new data sample is mapped to *F* at each time. Based on the above analysis, the following equation can be obtained:

(6) $$\begin{array}{c} G\left(f,t+\Delta T\right)\leq \underset{x\in s\left(f,t\right)}{\sum }g\left(x,t+\Delta T\right)+\sum_{t=0}^{\Delta T-1}2^{-\delta i}\\ =\sum_{x\in s\left(f,t\right)}2^{-\delta \Delta T}g\left(x,t\right)+\frac{1-2^{-\delta \Delta T}}{1-2^{-\delta }}\\ =2^{-\delta \Delta T}G\left(x,t\right)+\frac{1-2^{-\delta \Delta T}}{1-2^{-\delta }}. \end{array}$$

Suppose

(7) $$\begin{array}{c} 2^{-\delta \Delta T}G\left(x,t\right)+\frac{1-2^{-\delta \Delta T}}{1-2^{-\delta }}=\sigma , \end{array}$$

can get

(8) $$\begin{array}{c} 2^{-\delta \Delta T}=\frac{S\left(x,t\right)\left(1-2^{-\delta }\right)-1}{\sigma \left(1-2^{-\delta }\right)-1}. \end{array}$$

The density detection period should take the minimum integer value between Δ*T*_min_^−^ and Δ*T*_min_^+^. According to Theorems 1 and 2, the following (3) was worked out:

(9) $$\begin{array}{c} P=\left\lfloor \min\left\{\frac{1}{\gamma }\log\frac{\delta }{\delta -1},\left|\frac{1}{\gamma }\log\frac{G\left(x,t\right)\left(1-2^{-\delta }\right)-1}{\delta \left(1-2^{-\delta }\right)-1}\right|\right\}\right\rfloor . \end{array}$$

**Theorem 3 .**

When the parameter is greater than a certain critical value, the sparse grid cannot be upgraded to the dense grid.

It is proved that the sum of densities of data sample points in the set *S*(*f*, *t*) at time *t* is ∑_*x*∈*S*(*f*, *t*)_*g*(*x*, *t*), and the sum of densities at time *t*+Δ*T* is ∑_*x*∈*s*(*f*, *t*)_*g*(*x*, *t*+Δ*T*). If the decreasing speed of the sum of density of data sample points in the set *S*(*f*, *t*) is greater than the increasing speed of the sum of density of all newly arrived data samples within Δ*T* time interval, then the sparse grid *f* cannot be upgraded to a dense grid, and the equation is as follows:

(10) $$\begin{array}{c} \sum_{x\in s\left(f,t\right)}g\left(x,t\right)-\sum_{x\in s\left(f,t\right)}g\left(x,t+\Delta T\right)>\sum_{t=0}^{\Delta T-1}2^{-\delta i}. \end{array}$$

Calculate

(14) $$\begin{array}{c} \left(1-2^{-\delta \Delta T}\right)g\left(x,t\right)>\frac{1-2^{-\delta \Delta T}}{1-2^{-\delta }},\\ \delta >\;\log\frac{G\left(x,t\right)}{G\left(x,t\right)-1}. \end{array}$$

According to Theorem 3, when the parameter *δ* satisfies *δ* > log*G*(*x*, *t*)/*G*(*x*, *t*) − 1, where *G*(*f*, *t*) represents the density of sparse grid unit *f* at time *t*, grid unit *f* will not be upgraded to dense grid.

### 2.6. Simulation Experiment and Performance Evaluation under the Density-Grid Clustering Algorithm

In this study, the performance of the density-grid clustering algorithm was verified through the experiment, and it was compared with the single density-based clustering algorithm and the single grid-based clustering algorithm. The hardware platform used in the experiment was a personal computer with Intel® Core^(TM)^ i3-2100 3.10GH central processing unit (CPU) and 4 GB random access memory (RAM). The software environment adopted Visual Studio 2020 and MATLAB R2008a. The experimental parameters were set as *δ* = 2.5 and *γ* = 0.24. In the data set in this experiment, each data sample had 40 attributes, of which 32 continuous attributes constituted a subdata set. For the more accurate experimental results, the data used were standardized before the experiment.

The clustering effects of the three algorithms were evaluated by the purity and the entropy.

The calculation method of cluster purity is as follows:

(12) $$\begin{array}{c} \text{cluster purity}=\frac{\sum_{i}^{N}\left|{\text{M}}_{i}^{h}\right|/\left|{\text{M}}_{i}\right|}{N}\times 100\text{\%}. \end{array}$$

In (12), *N* represents the number of classes in the clustering result, |M_*i*_^*h*^| represents the number of all cluster labels in the *i*th cluster, and |M_*i*_| represents the data of the data in the *i*th cluster. The higher the purity of the cluster, the more similar the data in the cluster, and the greater the similarity between the data.

The calculation method of clustering entropy is as follows:

(13) $$\begin{array}{c} \text{clustering entropy}=\sum_{i}^{N}\sum_{x\in M_{i}}I^{2}\left(x,p_{i}\right). \end{array}$$

In (13), *M*_*i*_ represents the number of all data in the *i*th cluster, and *I*^2^(*x*, *p*_*i*_) represents the distance from data *x* to the center of the cluster *p* to which it belongs. The smaller the clustering entropy, the higher the clustering degree of data in the cluster, and the better the clustering quality. The higher the clustering entropy, the more scattered the data in the cluster, and the lower the clustering quality.

### 2.7. Construction Methods and Contents of the Performance Evaluation Indicator System

Key performance indicators referred to that after an organization analysed the characteristics of individual work performance; the indicators that represented the performance best were taken as key indicators for performance evaluation [27]. The balanced scorecard mainly emphasized that there was a balance between various indicators. Because of its simple and reasonable evaluation indicators and weight design, it is easy to operate in use and the most widely used in the performance evaluation of major enterprises and organizations [28]. The stakeholder theory explained the core of business management and performance assessment in details and provided a theoretical basis for performance evaluation [29]. The stakeholder theory was introduced as the main research method in this study, and key performance indicators and balanced scorecard were the auxiliary methods to construct a performance evaluation indicator system.

Any performance evaluation tool had its advantages and disadvantages. When choosing an evaluation tool, it should be considered whether it met the organization's own conditions. Various evaluation tools were widely used in the performance evaluation of hospital economic management, but they did not form a comprehensive and unified evaluation mode. The performance evaluation indicators of well-defined hospital economic management were listed out one by one, to obtain the best evaluation indicators as candidate indicators, with integrity, relevance, countability, and independence as the attribute principles for selection. The questionnaire was designed based on the Mitchell scoring method mainly in this study, and these selected candidate indicators were taken as the source of performance evaluation indicators of public hospital economic management. Then, the Delphi method was adopted to determine the final evaluation indicators and their weights.

### 2.8. Research Process and Quality Control

Mitchell scoring method scores stakeholders from three aspects: legitimacy, power, and urgency. According to the scoring results, stakeholders are divided into three types: decisive stakeholders, that is, they have three attributes: legitimacy, power, and urgency. Stakeholders of this type are the first objects that organizations pay close attention to and contact. Expected stakeholders are with any two of the above attributes; potential stakeholders have one of the above three attributes. Mitchell scoring method optimizes the limitations of multicone subdivision method, which makes the classification of stakeholders more scientific and easier to operate. According to the Mitchell scoring method, the expert consultation form for the performance evaluation indicator system of hospital economic management was designed with the candidate indicators. The survey objects of the expert consultation form were mainly health administration staff, medical college tutors, technologists in hospital, hospital management personnel, and hospital financial management personnel. The candidate indicators belonging to the performance evaluation indicators of hospital economic management were scored in entitlement, legitimacy, and urgency. The total score was 5 points, which indicated the strongest entitlement, legitimacy, and urgency, while 1 point suggested the weakest. Then, the weights of the indicators were obtained according to the results of expert consultation questionnaire survey.

Delphi method is based on the professional knowledge, experience, and subjective judgment ability of many experts and is especially suitable for analysis that lacks information and historical data and is influenced by many other factors. Among them, the survey consultation form uses the anonymity of experts, and the consultation experts only contact with the investigators, and there is no horizontal contact between the experts, which can well avoid the interference of experts on the results and reflect the real thoughts of experts. The Delphi method was used for the quality control of the experts participating in the scoring, aiming to ensure the quality of the expert consultation form. The prescribed procedures were strictly followed, and independent consultations of each expert were carried out. Experts finished the questionnaire surveys in strict accordance with the procedures to fully guarantee the scoring. After multiple questionnaire surveys, the expert opinions were collected, and finally the performance evaluation indicator system was formed. The system of hospital economic management was divided in the importance, mainly including core indicators, potential indicators, and marginal indicators, and the weights of relevant indicators were determined finally.

### 2.9. General Information of Experts

16 experts from the practical and academic fields related to hospital economic management were invited to participate in the performance evaluation of hospital economic management. They were from health administration, medical colleges, hospital technologies, hospital management, and hospital financial management.

Table 1 shows the general information of the experts. In the first round of consultation, there were 9 experts (56.25%) who were 35–55 years old, accounting for the most of all experts. 7 experts (43.75%) were graduated with a master degree, which was the most; and there was no junior college graduate. It was proved that the experts had the high cultural literacy with a great understanding of the contents in consultation form. There were 13 experts (52.25%) with deputy senior titles or above, and 13 experts (81.25%) had worked for more than 10 years. 1 (6.25%), 6 (37.50%), 3 (18.75%), 4 (25.00%), and 2 (12.50%) experts were working in the health administration, medical colleges, medical technologies, hospital management, and hospital financial management, respectively. In the types of the work units, the distribution of experts was relatively reasonable. These experts were all capable in the actual work so that they could contact and deal with problems as soon as they encountered.

Two rounds of expert questionnaire surveys were conducted in this study. The survey content includes the importance and feasibility evaluation of indicators at all levels, comparison score, modification, and supplementary opinions on the importance of indicators at the same level. The response rates of the two rounds of questionnaire surveys were 100%, indicating that the experts were highly motivated to participate in and concern about the study.

### 2.10. Coordination Degree of Expert Opinions

The coordination degree of expert opinions referred to the degree of disagreement among experts on the stakeholder evaluation indicator scoring in entitlement, legitimacy, and urgency. It was assumed that C represented the coordination coefficient, and the value range of C was [0, 1]. The larger the value of C, the better the coordination degree of expert opinions on the stakeholder evaluation indicator scoring. If the coordination coefficient C was different after check, it meant a good coordination degree of expert opinions and the result was advisable; otherwise, it was unadvisable.

## 3. Results and Discussion

### 3.1. Comparison Results of Simulation Experiment

Figure 4 shows the comparison of the purity, entropy, and memory consumption of three clustering algorithms. In this section, real data sets are used to test and compare network-based clustering algorithm, density-based clustering algorithm, and network density-based clustering algorithm. The parameter setting data flow rate *v* = 1000, and other parameters are the same as those in the dynamic evolution operation experiment of data stream. With the density-grid clustering algorithm, the parameter *γ* could be compared with the grid density. Then, the density detection period was selected adaptively, which could capture the changes of the data flow at any time. The results showed that, compared with simple network clustering algorithm and density clustering algorithm, the clustering algorithm based on density network produces higher purity (94% VS 73% VS 67%) and lower entropy (0.9 VS 1.4 VS 1.54), which effectively saved memory consumption, and the difference is statistically significant (*P* < 0.05).

The density-based clustering algorithm mainly dealt with static data sets. Lee et al. [30] found that the algorithm could search for clusters in different shapes and then process the noise in the data set effectively. The grid-based clustering algorithm mainly dealt with the multiresolutions. He et al. [31] illustrated that the algorithm could classify the data set space, which was dispersed into some units and formed a grid shape gradually. Then, all clustering operations were performed on the grid. The major advantages of the grid-based algorithm were the short time and fast speed for processing the data sets. In this study, the two clustering algorithms were integrated into the density-grid clustering algorithm, and then the data flow was clustered. It turned out that the data flow sample space could be divided into many small grids, and each data sample in the data flow was mapped to a corresponding small grid. Then, the data flow sample was clustered through the density of these grids. In addition, the density-grid clustering algorithm was also optimized in its density detection period of grid cells and sparse grid detection.

### 3.2. Construction Results of Performance Evaluation Indicator System

With two rounds of expert consultation questionnaire surveys, the performance evaluation indicator system of hospital economic management was finally established. There were 6 first-level indicators, namely, budget management, financial fund management, cost control, medical expense management, medical efficiency, and medical quality, respectively. There were also 25 second-level indicators, which are shown in Figure 5 in details.

### 3.3. Classification Results of Performance Evaluation Indicators

According to the Mitchell's scoring method, the performance evaluation indicators were classified in three dimensions of entitlement, legitimacy, and urgency.

Entitlement referred to the indictors directly related to the status and capability of hospital economic management. As shown in Figure 6, the larger the score, the greater the influence on the hospital, while the smaller the score, the slighter the influence.

The indicators that had a greater influence on the hospital economic management were listed as follows with the score greater than 4.5 points. The second-level indicators in the first-level budget management included the budget revenue implementation efficiency (4.91 points), the budget expenditure implementation efficiency (4.85 points), and the implementation efficiency of special appropriation (4.89 points). In financial fund management, the second-level indicators above 4.5 points were balance ratio of payments (4.52 points) and asset-liability ratio (4.67 points). In cost control, outpatient service income cost rate (4.52 points) was included. In medical expense management, those consisted of the medical insurance accounting rate (4.65 points), the average cost of discharged patients per time (4.52 points), the average cost of outpatient emergency per visit (4.58 points), the drug expenditure ratio (4.78 points), and the consumables ratio (4.63 points).

With the score between 4 and 4.5 points, the following indicators had the moderate influence on hospital economic management. In financial fund management, the liquidity ratio (4.12 points) was on the list. In cost control, inventory turnover ratio (4.31 points), hospitalization income cost rate (4.35 points), and consumption of drugs and health consumables in 100 RMB income (4.34 points) were included. In medical efficiency, outpatient emergency visits (4.39 points), number of discharged patients (4.32 points), number of surgeries (4.31 points), average length of stay (4.42 points), and utilization rate of beds (4.32 points) were all in this score range. In medical quality, coincidence of admission and discharge diagnoses (4.12 points), coincidence of preoperative and postoperative diagnoses (4.05 points), and recovery rate of inpatients (4.04 points) were also included.

Only accounts receivable turnover days (3.78 points) and depreciation period of fixed assets (3.95 points) had the score less than 4 points, as well as little influence on hospital economic management.

Legitimacy referred to the influence of some indicators in legal benefits, morality, or special hospital economic management. The larger the score, the higher the legitimacy of an indicator. It could be observed in Figure 7 for details.

The indicators, with the score more than 4.5 points and high legitimacy, were listed as follows. In the first-level indicator budget management, all of the budget revenue implementation efficiency (4.91 points), budget expenditure implementation efficiency (4.86 points), and implementation efficiency of special appropriation (4.78 points) met the situation. In financial fund management, only asset-liability ratio (4.92 points) was listed. In cost control, outpatient service income cost ratio (4.67 points), hospitalization income cost ratio (4.85 points), and consumption of drugs and health consumables in 100 RMB income (4.82 points) were included. In medical expense management and medical efficiency, medical insurance accounting rate (4.87 points), average cost of discharged patients per time (4.67 points), average cost of outpatient emergency per visit (4.86 points), drug expenditure ratio (4.62 points), and outpatient emergency visits (4.75 points) were on the list.

The indicators with the score between 4 and 4.5 points had a moderate legitimacy. In financial fund management, balance ratio of payments (4.43 points) and liquidity ratio (4.24 points) were in the range. In cost control, depreciation period of fixed assets (4.32 points) and inventory turnover ratio (4.25 points) were also included in the range. In medical efficiency, outpatient emergency visits (4.25 points), number of discharged patients (4.27 points), number of surgeries (4.26 points), average length of stay (4.35 points), and utilization rate of beds (4.41 points) were listed. In medical quality, all of the coincidence of admission and discharge diagnoses (4.36 points), coincidence of preoperative and postoperative diagnoses (4.25 points), and recovery rate of inpatients (4.12 points) went with the moderate legitimacy as well.

The indicators with less legitimacy had a score below 4 points, including the accounts receivable turnover days (3.87 points) only.

Urgency referred to whether the indicators could attract attention of the hospital and related administrative department managers immediately. The larger the score, the stronger the urgency; and the scores of various second-level indicators are shown in Figure 8.

As the score was above 4.5 points, the indicators had a greater urgency. Such second-level indicators included budget revenue implementation efficiency (4.67 points), budget expenditure implementation efficiency (4.58 points), and implementation efficiency of special appropriation (4.75 points) in the first-level indicator budget management. The medical insurance accounting rate (4.81 points) and the drug expenditure ratio (4.71 points) in medical expense management were also included.

Scored 4–4.5 points, the indicators had a moderate urgency. In financial fund management, the balance ratio of payments was 4.35 points, and the asset-liability ratio was 4.37 points. In cost control, outpatient service income cost rate, hospitalization income cost rate, and consumption of drugs and health consumables in 100 RMB income were 4.12 points, 4.26 points, and 4.41 points, respectively. In medical expense management, the average cost of discharged patients per time (4.35 points), the average cost of outpatient emergency per visit (4.41 points), and the consumables ratio (4.23 points) were on the list. In medical efficiency, all of the outpatient emergency visits (4.35 points), the number of discharged patients (4.37 points), the number of surgeries (4.41 points), average length of stay (4.28 points), and utilization rate of beds (4.36 points) were in this range. Besides, coincidence of admission and discharge diagnoses in medical quality reached 4.3 points.

Liquidity ratio (3.78 points), accounts receivable turnover days (3.56 points), depreciation period of fixed assets (3.86 points), inventory turnover ratio (3.95 points), coincidence of preoperative and postoperative diagnoses (3.78 points), and recovery rate of inpatients (3.76 points) had a less urgency with the score less than 4 points.

According to the classification of stakeholder theory, those with scores above two dimensions (including two dimensions) above 4.5 points can be considered as core indicators, mainly including budget revenue implementation rate, budget expenditure implementation rate, financial special allocation implementation rate, asset-liability ratio, hospitalization revenue cost rate, medical insurance settlement rate, average cost of discharged patients, and drug proportion. If the score of more than two dimensions (including two dimensions) is more than 4 points, it can be considered as a potential index, mainly including business balance rate, current rate, depreciation period of fixed assets, outpatient income cost rate, consumption of sanitary consumables, consumables ratio, outpatient and emergency visits, discharge visits, operation visits, average hospitalization days, bed utilization rate, diagnosis coincidence rate of admission and discharge visits, diagnosis coincidence rate before and after operation, and hospitalization mixed cure and improvement rate. Those with more than two dimensions (including two dimensions) below 4 points can be considered as marginal indicators, including average collection period and inventory turnover rate.

The listed candidate indicators were evaluated from the three dimensions of entitlement, legitimacy, and urgency, aiming to determine whether the indicators should be taken into the performance evaluation indicator system of hospital economic management. 5 points represented the greatest entitlement, legality, and urgency, while 1 point meant the least. The numerical results of the entitlement, legality, and urgency were basically similar to the definition of comprehensive relevance scores. It was indicated that the scoring results in this study were more reliable, and it was more complete than the indicator system of Li and Hao (2018) [32].

### 3.4. Determination of the Weights of Performance Evaluation Indicators

6 first-level indicators with 25 second-level indicators were determined finally. The weights of the 6 first-level indicators are shown in Table 2, and those of the 25 second-level indicators are shown in Table 3.

After the determination of the performance evaluation indicators of hospital economic management, the Delphi method was used again for two rounds of expert consultation questionnaires of weighted indicators. With statistics on the standard deviation and mean of each indicator, it was finally determined that the coefficient of variation of first-level indicators was between 0.05 and 0.14 and that of second-level indicators was in the range of 0.05–0.15. It was suggested that experts gave the higher credibility in scoring the weights of indicators after two rounds of questionnaires. The total score of weight was 100 points in this study; but actually, it was calculated as a percentage. Therefore, the indicator system could be used for comparative research, which was slightly different from the research of Wei et al. [33].

There was a strong economic management performance of this study itself. In the process of constructing the performance evaluation indicator system, special attention was paid to the orientation of economic indicators. The ultimate goal of the performance evaluation was to optimize the hospital running efficiency and enhance the hospital's role in improving health of people, which reflected the social responsibility that the hospital should be born. Although a relatively complete and practical performance evaluation indicator system of hospital economic management was proposed, it remained at the level of theoretical inquiry for some indicators without being tested and verified by comprehensive practice. Therefore, it needed to be further explored in related fields, especially in practical management.

## 4. Conclusion

The framework of the electronic health management system was designed in this study under the density-grid clustering algorithm. Meanwhile, the included candidate indicators were taken to design the expert questionnaire for the performance evaluation indicator system of hospital economic management. With the Delphi method, 16 experts in related fields and hospital administration were chosen for the questionnaire survey, which was to evaluate the included candidate indicators in entitlement, legitimacy, and urgency. After two rounds of expert questionnaire surveys, the weight of each indicator in the system was determined. The density-grid clustering algorithm gave higher purity and lower entropy, which saved memory massively. 6 first-level indicators were finally brought into the performance evaluation indicator system of hospital economic management, including budget management, financial fund management, cost control, medical expense management, medical efficiency, and medical quality. There were also 25 second-level indicators affiliated to the first-level indicators who were ascertained. In budget management, there were budget revenue implementation efficiency, budget expenditure implementation efficiency, and implementation efficiency of special appropriation. In financial fund management, there were balance ratio of payments, asset-liability ratio, liquidity ratio, and accounts receivable turnover days. Cost control was composed of depreciation period of fixed assets, inventory turnover ratio, outpatient service income cost rate, hospitalization income cost rate, and consumption of drugs. In medical expense management, the medical insurance accounting rate, average cost of discharged patients per time, average cost of outpatient emergency per visit, drug expenditure ratio, and consumables ratio were included. Medical efficiency consisted of the outpatient emergency visits, number of discharged patients, number of surgeries, average length of stay, and utilization rate of beds. Medical quality was made up of the coincidence of admission and discharge diagnoses, the coincidence of preoperative and postoperative diagnoses, and the recovery rate of inpatients. The results of the two following rounds of expert consultation questionnaires found that the scoring of indicator weights by experts were highly credible. The deficiency of this study lies in the fact that the indicators are screened in combination with the background of big data, which may lead to the imperfect index system. Therefore, it is necessary to broaden the field of evaluation indicators in the later period to meet the needs of performance evaluation of hospital economic management in China.

## Figures and Tables

**Figure 1:** Basic architecture of the electronic health management platform.

**Figure 2:** Framework diagram of the electronic health management system based on business processes.

**Figure 3:** Construction process of electronic health management index system.

**Figure 4:** Comparison of purity, entropy, and memory consumption of the three algorithms. (a) Clustering purity comparison. (b) Clustering entropy comparison. (c) Memory consumption comparison. ∗ indicates the differences statistically significant compared with results of the density-grid clustering algorithm (*P* < 0.05).

**Figure 5:** Performance evaluation index system of hospital economic management.

**Figure 6:** Entitlement evaluation of second-level indicators. (a) Entitlement evaluation of second-level indicators in budget management and financial fund management; (b) entitlement evaluation in cost control and medical expense management; (c) entitlement evaluation in medical efficiency and medical quality.

**Figure 7:** Legitimacy evaluation of second-level indicators. (a) Legitimacy evaluation of second-level indicators in budget management and financial fund management; (b) legitimacy evaluation in cost control and medical expense management; (c) legitimacy evaluation in medical efficiency and medical quality.

**Figure 8:** Urgency evaluation of second-level indicators. (a) Urgency evaluation of second-level indicators in budget management and financial fund management; (b) urgency evaluation in cost control and medical expense management; (c) urgency evaluation in medical efficiency and medical quality.

**Table 1:** General information of experts.

Items	Classification	Number (proportion)
Age	<35 years old	3 (18.75%)
	35–55 years old	9 (56.25%)
	≥56 years old	4 (25.00%)

Highest education qualification	Doctor	6 (37.50%)
	Master	7 (43.75%)
	Bachelor	3 (18.75%)

Professional title	Junior	0 (0.00%)
	Medium grade	3 (18.75%)
	Deputy senior	8 (20.00%)
	Senior	5 (31.25%)

Type of work unit	Health administration	1 (6.25%)
	Medical colleges	6 (37.50%)
	Medical technologies	3 (18.75%)
	Hospital management	4 (25.00%)
	Hospital financial management	2 (12.50%)

Working years	<10 years	3 (18.75%)
	10–20 years	2 (12.50%)
	20–30 years	5 (31.25%)
	>30 years	6 (37.50%)

Regent's canal	Completely unfamiliar	0 (0.00%)
	Basically unfamiliar	0 (0.00%)

Familiarity of hospital management	Generally familiar	1 (6.25%)
	Relatively familiar	6 (37.50%)
	Very familiar	9 (56.25%)

**Table 2:** Weights of first-level indicators.

First-level indicators	Indicator number	Indicated number	Standard deviation	Mean	Coefficient of variation	Weight
Budget management	A	1	1.26	16.89	0.12	16.9
Financial fund management	B	2	1.36	17.37	0.05	17.4
Cost control	C	3	2.16	15.44	0.13	15.4
Medical expense management	D	4	2.28	13.58	0.08	13.6
Medical efficiency	E	5	1.45	15.37	0.14	15.4
Medical quality	F	6	2.26	21.35	0.07	21.3
Total score						100 points

**Table 3:** Weights of second-level indicators.

Second-level indicators	Indicator number	Indicated number	Units	Standard deviation	Mean	Coefficient of variation	Weight
Budget revenue implementation efficiency	A1	1	%	1.56	8.61	0.15	8.6
Budget expenditure implementation efficiency	A2	2	%	1.52	1.12	0.09	1.1
Implementation efficiency of special appropriation	A3	3	%	1.78	7.23	0.12	7.2
Balance ratio of payments	B1	4	%	2.56	3.71	0.08	3.7
Asset-liability ratio	B2	5	%	2.78	3.72	0.11	5.3
Liquidity ratio	B3	6	%	2.45	2.83	0.13	2.8
Accounts receivable turnover days	B4	7	Day	2.67	5.61	0.16	5.6
Depreciation period of fixed assets	C1	8	Year	2.67	5.62	0.14	2.9
Inventory turnover ratio	C2	9	%	2.43	3.63	0.08	3.6
Outpatient service income cost rate	C3	10	%	1.71	3.71	0.05	3.7
Hospitalization income cost rate	C4	11	%	2.56	2.52	0.07	2.5
Consumption of drugs and health consumables in 100 RMB income	C5	12	RMB	1.89	2.73	0.13	2.7
Medical insurance accounting rate	D1	13	%	1.45	3.39	0.12	3.4
Average cost of discharged patients per time	D2	14	RMB	1.23	2.08	0.07	2.1
Average cost of outpatient emergency per visit	D3	15	RMB	2.45	2.07	0.13	2.7
Drug expenditure ratio	D4	16	%	2.67	3.09	0.08	3.1
Consumables ratio	D	17	%	1.89	2.28	0.12	2.3
Outpatient emergency visits	E1	18	Case	1.12	2.47	0.16	2.5
Number of discharged patients	E2	19	Case	2.13	4.09	0.07	4.1
Number of surgeries	E3	20	Case	2.14	2.68	0.06	2.7
Average length of stay	E4	21	Day	2.67	3.77	0.14	3.8
Utilization rate of beds	E5	22	%	1.81	2.25	0.07	2.3
Coincidence of admission and discharge diagnoses	F1	23	%	2.86	7.21	0.08	7.3
Coincidence of preoperative and postoperative diagnoses	F2	24	%	1.57	5.75	0.15	5.8
Recovery rate of inpatients	F3	25	%	2.89	8.16	0.09	8.2
Total score							100 points

## Data Availability

All data included in this study are available upon request by contact with the corresponding authors.
